# Overexpression of miRNA-93-5p Promotes Proliferation and Migration of Bladder Urothelial Carcinoma via Inhibition of KLF9

**DOI:** 10.1155/2022/8911343

**Published:** 2022-03-09

**Authors:** Tao Li, Qingjiang Xu, Yongbao Wei, Rongcheng Lin, Zhiwei Hong, Rong Zeng, Weilie Hu, Xiang Wu

**Affiliations:** ^1^Provincial Clinical Medical College of Fujian Medical University, Fuzhou 350001, China; ^2^Department of Urology, Fujian Provincial Hospital, Fuzhou 350001, China; ^3^Department of Urology, Guangdong Hydropower Hospital, Guangzhou 511340, China

## Abstract

We focused on studying the effects of a key miRNA-mRNA axis in bladder urothelial carcinoma (BUC). Firstly, miRNAs and mRNAs differentially expressed in BUC were analyzed. Clinical information in the TCGA database was used for survival analysis, and the regulator of miRNA-93-5p was predicted. miRNA-93-5p and KLF9 mRNA expression were detected by qRT-PCR. Protein level detection and targeting measurement were, respectively, achieved by western blot and dual-luciferase approaches. The proliferative, invasive, and migratory abilities were tested through CCK-8, Transwell, and wound healing methods. Cell apoptosis in each group was detected through flow cytometry. As discovered, miRNA-93-5p level was markedly high in BUC cells while KLF9 expression was remarkably low. miRNA-93-5p overexpression promoted BUC cell abilities. Besides, miRNA-93-5p inhibited KLF9 expression. Furthermore, KLF9 overexpression dramatically attenuated such promotion on cancer cell abilities. On the whole, miRNA-93-5p/KLF9 axis facilitated BUC progression, offering a new potential target for BUC patients.

## 1. Introduction

Bladder cancer (BC), a prevalent tumor in the urogenital system, is caused by the overgrowth of bladder mucosa epithelial cells, with high morbidity and low 5-year survival rate [1]. Approximately 34% of patients die of metastatic BC [2]. An estimated 61,700 patients in the United States were diagnosed with BC, and 12,870 died of the disease in 2019 [3]. Bladder urothelial carcinoma (BUC) accounts for 90% of all BC cases and displays a high relapse rate [4, 5]. Local invasion and metastasis to distant organs (lung, liver, and bone) contribute to deaths pertinent to BUC [6]. So far, BUC complicated with tumor metastasis remains unresolved. Therefore, to deeply research the underlying molecular mechanism of metastasis and invasion of BUC is essential, thereby providing a novel therapeutic target and increasing patient's survival rate.

Studies illustrated that miRNAs are closely relevant to tumor occurrence and work as a cancer inhibitor or promoter [7] to be involved in tumor cell differentiation, growth, and apoptosis [8]. Therefore, miRNAs can be used as diagnostic and prognostic biomarkers. miRNA-93-5p researched in this study, as one of the most common reported circulating miRNAs, is located in chromosome 11q22.1 and originates from the miR-106b-25 family [9]. Among studies of tumor-related miRNAs, miRNA-93-5p was found to be a reference gene of colorectal cancer [10] and vulvar squamous carcinoma [11]. Besides, studies demonstrated that miRNA-93-5p expression level is abnormally elevated in ovarian cancer [12] and prostate cancer [13]. A study reported that miRNA-93-5p is ectopically at a high level in breast cancer [14]. Nevertheless, little is known about the downstream modulatory mechanism of miRNA-93-5p in the BUC progression.

Kruppel-like factors (KLFs) are transcription factors widely involved in cell activity and embryonic development [15]. One study presented that KLF9, a member of the KLF family, participates in dexamethasone-induced macrophage apoptosis through mitochondrial-dependent apoptosis [16]. Currently, little is reported about KLF9 as a cancer regulator. A study reported that methylated KLF9 is an independent prognostic factor of breast cancer [17]. miRNA-940 facilitates glioma cell invasion and proliferation by mediating KLF9 [18]. Nevertheless, the mechanism of KLF9 in BUC is unclear. Therefore, researching the regulation of KLF9 on BUC is helpful for finding a novel prognostic biomarker and developing a new therapeutic method.

This work illustrated that miRNA-93-5p was stimulated in BUC and bound KLF9 to aggravate BUC. These results demonstrated the critical impacts miRNA-93-5p performed on BUC.

## 2. Materials and Methods

### 2.1. Data Availability

htseq-count data (tumor: 408; normal: 19) and Isoform Expression Quantification data (tumor: 412; normal: 19) related to BUC were accessed from the TCGA Bladder Urothelial Carcinoma (BLCA) dataset. Afterward, differential analysis was undertaken on htseq-count data and Isoform Expression Quantification data by using the R package “edgeR,” with ∣logFC | >2, adj.*p* value < 0.05 as screening standard for differential miRNAs and normal samples as the control. Next, the targets of miRNA-93-5p were predicted with starBase, TargetScan, miRDB, miRTarBase, and miRanda databases. The predicted mRNAs were intersected with downregulated mRNAs (∣logFC | >2) to obtain candidate regulatory mRNAs of miRNA-93-5p.

### 2.2. Cell Lines and Cell Culture

Immortalized human normal uroepithelial cell line SV-HUC-1 was cultured in CM7-1medium (HyClone, USA). Human BUC cell line BT-B was cultivated in Dulbecco's Modified Eagle's Medium-High Glucose (DMEM-H, Gibco, USA). BUC cell lines RT4 and RT-112 were cultured in CM5-1 medium (HyClone, USA). BUC cell line 5637 was placed in CM2-1 medium (HyClone, USA). Cell lines used in the experiments are shown in Table 1. All cells were cultured at 37°C with 5% CO_2_.

### 2.3. Cell Transfection

miRNA-93-5p mimics (miR-mimics), negative control mimics (miR-NC), pcDNA3.1-KLF9 plasmids encoding KLF9 (oe-KLF9), and blank pcDNA3.1 plasmids (oe-NC) were bought from RiboBio (Guangzhou, China). The Lipofectamine 2000 kit (Invitrogen, USA) was applied to transfect miR-mimics, miR-NC, or target plasmids into cancer cell lines.

### 2.4. Real-Time Quantitative Fluorescence Polymerase Chain Reaction (qRT-PCR)

Total RNA was separated from cells by using the TRIzol kit (Life Technologies, USA). Total RNA concentration was determined by the NanoDrop 2000 system (Thermo Fisher Scientific, USA). Afterward, miRNAs extracted from cells were reversely transcribed into cDNA through the TaqMan®reverse transcription kit (Applied Biosystems, USA). Next, mRNAs were reversely transcribed into cDNA with PrimeScript RT Master Mix (Takara, Japan). Thereafter, miRNA and mRNA expression levels were measured by the miScript SYBR Green PCR Kit (Qiagen, Germany) and SYBR® Premix Ex Taq TM II (Takara, Japan), respectively. qRT-PCR was conducted on Applied Biosystems® 7500 Real-Time PCR Systems (Thermo Fisher Scientific, USA) to detect miRNA-93-5p and KLF9 mRNA expression levels. GAPDH and U6 were taken as internal references for KLF9 and miRNA-93-5p, respectively. The 2^-*ΔΔ*Ct^ value was used to calculate the relative expression of miRNA-93-5p and KLF9 mRNA in different treatment groups. Primer sequences are shown in Table 2.

### 2.5. Western Blot Assay

Protein extraction was performed using RIPA lysis buffer (Beyotime, China), and concentration was determined with the BCA kit (Thermo Fisher Scientific, USA). Equivalent proteins (20 *μ*g) of each group were transferred onto a polyvinylidene fluoride membrane after sodium dodecyl sulfate-polyacrylamide gel electrophoresis. Next, the membrane was blocked with 5% bovine serum albumin (BSA) and then reacted with primary antibodies at 4°C overnight. Afterward, the membrane was incubated with secondary antibodies for 2 h. Protein blots were observed by enhanced chemiluminescence (ECL) (GE Healthcare, USA) and quantified by a Quantum One System Image Analyzer (Bio-Rad, USA). Antibodies used in the experiment were primary antibodies rabbit anti-KLF9 (ab227920, 1 : 2000), rabbit anti-p-JAK1 (ab203784,1 : 1000), rabbit anti-JAK1 (ab133666,1 : 1000), rabbit anti-p-STAT3 (ab76315,1 : 2000), rabbit anti-STAT3 (ab68153,1 : 1000), rabbit anti-GAPDH (ab181602, 1 : 10000), and secondary antibody goat anti-rabbit IgG (ab205718, 1 : 10000). These antibodies were purchased from Abcam (UK).

### 2.6. Cell Proliferation Evaluation

Cell proliferative ability was evaluated by using the Cell Counting Kit-8 (CCK-8) (Dojindo, Japan). Cells were inoculated in 96-well plates (2 × 10^4^ cells/well) and cultured with 5% CO_2_ at 37°C. 0, 24, 48, 72, and 96 h later, 10 *μ*L CCK-8 reagent was supplemented. Afterward, cells were cultured with 5% CO_2_ at 37°C for another 2 h. Absorbance at 450 nm wavelength was read by a microplate reader (Thermo Fisher Scientific, USA).

### 2.7. Cell Invasion Assay

Cells (5 × 10^4^ cells/well) were added into the Transwell chamber coated with Matrigel (8 *μ*M; Biosciences, USA). DMEM containing 10% FBS was added into the lower chamber. 24 h later, cells in the upper chamber were removed gently. Afterward, invading cells in the lower chamber were treated with 4% paraformaldehyde overnight and 0.1% crystal violet. Images were taken by an optical microscope. Invading cells were counted in 3 random fields.

### 2.8. Wound Healing Assay

Cells were inoculated into 6-well plates (1 × 10^5^ cells/well) until a single layer of fused cells was formed. A 200 *μ*L sterile micropipette tip was employed to gently scrape through the center of the single layer to create a wound (about 0.5 mm). Afterward, cells were washed with PBS twice to remove separated cells. Then, cells were cultured in a serum-free medium. Images at 0 and 24 h were captured under an inverted microscope (Olympus, Japan). Wound width was measured through ImageJ software (NIH, USA), and wound healing percentage was calculated as (wound healing percentage = (width at 0 h − width at 24 h)/width at 0 h).

### 2.9. Dual-Luciferase Detection

pmiRGLO luciferase reporter gene vectors (Promega, USA) of wild-type (WT) and mutant (MUT) KLF9 3′-UTR were constructed. Afterward, BUC cell line RT4 was seeded into 96-well plates (3 × 10^5^), and then, 100 nM miR-mimics/miR-NC and KLF9-WT/KLF9-MUT plasmids were cotransfected into cells by utilizing Lipofectamine 2000. After 48 h of culture, luciferase activity was detected through a dual-luciferase reporter gene detection system (Promega, USA).

### 2.10. Cell Apoptosis Detection

Cell apoptotic ability was assayed by Annexin V-fluorescein isothiocyanate (FITC) cell apoptosis detection kit. Collected cells were suspended in 300 *μ*L binding buffer and then incubated with 5 *μ*L Annexin V-FITC solution at 4°C for 30 min. Afterward, 5 *μ*L propidium iodide (PI, Sigma, USA) was used for further incubation for 5 min. Lastly, cell apoptosis was examined and analyzed with BD FACSCanto II equipped with BD FACSDiva software (Becton-Dickinson, USA).

### 2.11. Statistical Analysis

Each assay underwent no less than three repetitions. Data analysis was performed on GraphPad Prism 6.0 (La Jolla, CA). Outcomes were displayed as mean ± standard deviation. Significant difference was analyzed by Student's *t-*test or one-way analysis of variance. Pearson correlation analysis was used for analyzing correlation. Statistical significance was shown when *p* values < 0.05.

## 3. Results

### 3.1. miRNA-93-5p Level Is Remarkably Upregulated in BUC

144 differential miRNAs were obtained (Figure 1(a)). Bioinformatics analysis in TCGA-BLCA exhibited remarkably stimulated miRNA-93-5p in BUC tissue (Figure 1(b)). Meanwhile, a study confirmed such upregulation in BC [19]; therefore, miRNA-93-5p was chosen for research. Thereafter, qRT-PCR verified such upregulation at the cell level in BUC (Figure 1(c)). Overall, miRNA-93-5p was differentially activated in BUC.

### 3.2. miRNA-93-5p Overexpression Stimulates Malignant Functions of BUC Cells

As shown in Figure 1(c), miRNA-93-5pexpression was downregulated in BUC cell lines RT4 and RT-112; thus, these cells were taken for miRNA-93-5p overexpression. qRT-PCR displayed that miRNA-93-5p evidently enhanced after overexpression (Figure 2(a)). Afterward, the CCK-8 assay revealed that miRNA-93-5p overexpression noticeably stimulated BUC cell proliferative ability (Figure 2(b)). miRNA-93-5p overexpression notably hastened invasive and migratory capabilities of BUC cells (Figures 2(c) and 2(d)). Cell apoptosis assay manifested that miRNA-93-5p overexpression significantly downregulated the apoptotic level of BUC cells (Figure 2(e)). All the above results illustrated that miRNA-93-5p overexpression stimulated BUC cell malignant functions.

### 3.3. KLF9 Is Noticeably Downregulated in BUC Cells

Firstly, 1,595 differential mRNAs were screened by conducting differential analysis on mRNAs in the TCGA-BLCA dataset (Figure 3(a)). Afterward, the predicted target genes of miRNA-93-5p were intersected with downregulated mRNAs, and 9 differential mRNAs containing target binding sites of miRNA-93-5p were obtained (Figure 3(b)). Correlation analysis exhibited the highest correlation between miRNA-93-5p and KLF9 (Figures 3(c) and 3(d)). Hence, KLF9 was finally chosen for research. TCGA-BLCA data showed that KLF9 expression was conspicuously low in BUC tissue (Figure 3(e)). By qRT-PCR, KLF9 mRNA expression was markedly downregulated in BUC cell lines (Figure 3(f)). Likewise, western blot assay also unmasked a considerable drop of KLF9 protein expression in BUC cell lines than in normal cell line (Figure 3(g)). Hence, it was posited that KLF9 might be a target of miRNA-93-5p.

### 3.4. miRNA-93-5p Binds KLF9 in BUC

Database prediction discovered that miRNA-93-5p shared binding sites with KLF9 3′-UTR (Figure 4(a)). Based on the dual-luciferase method, miRNA-93-5p overexpression suppressed the luciferase activity of KLF9-WT 3′-UTR, whereas did not affect that of KLF9-MUT 3′-UTR (Figure 4(b)). Thereafter, qRT-PCR detected that miRNA-93-5p overexpression remarkably downregulated KLF9 mRNA expression in cells (Figure 4(c)). KLF9 protein level was significantly repressed after overexpressing miRNA-93-5p detected by western blot (Figure 4(d)). Overall, miRNA-93-5p downregulated KLF9 expression in BUC.

### 3.5. miRNA-93-5p Modulates BUC Cell Phenotypes via KLF9

To explore whether miRNA-93-5p could regulate BUC cells via targeting KLF9, we used RT4 and RT-112 cell lines to construct miR-NC+oe-NC, miR-NC+oe-KLF9, and miR-mimics+oe-KLF9. It was shown from qRT-PCR and western blot results that KLF9 mRNA and protein levels were considerably stimulated in the miR-NC+oe-KLF9 group, while those were comparatively decreased in the miR-mimics+oe-KLF9 group (Figures 5(a) and 5(b)), illustrating that miRNA-93-5p repressed KLF9. KLF9 overexpression remarkably constrained the viabilities of BUC, whereas such inhibition was diminished in the miR-mimics+oe-KLF9 group (Figure 5(c)). Afterward, it was found that the migratory and invasive abilities were significantly decreased after overexpressing KLF9. Nonetheless, the invasive and migratory abilities were remarkably increased and recovered in the miR-mimics+oe-KLF9 group compared with those in the oe-NC+oe-KLF9 group (Figures 5(d) and 5(e)). KLF9 overexpression hastened BUC cell apoptosis, while the effect was attenuated by overexpressing miRNA-93-5p (Figure 5(f)). The above results implied that miRNA-93-5p could accelerate cell phenotypes through downregulating KLF9 expression.

## 4. Discussion

Recently, a growing number of studies suggested the value miRNAs have in most cancers. A study demonstrated that miRNA-99a-5p targets mTOR to be a tumor inhibitor and enhances RAD001-induced human BUC cell apoptosis [20]. Decreased miRNA-199a-5p fosters BUC tumorigenesis through modulating the MLK3/NF-*κ*B pathway [21]. These miRNAs may be novel and potential biomarkers for BUC. Generally, miRNA-93-5p is considered a tumor promoter. For instance, miRNA-93-5p/IFNAR1 hastens endometrial carcinoma metastasis via the STAT3 pathway [9]. Highly conserved miRNA-93-5p has been recorded in vulvar squamous carcinoma [11] and colorectal cancer [10], whereas we demonstrated that miRNA-93-5p level was conspicuously upregulated in BUC through bioinformatics analysis and cell biological experiments. The reasons might be different genes that miRNA-93-5p mediated and different copy numbers. Moreover, cell functional experiments revealed that miRNA-93-5p overexpression accelerated BUC cell processes thereby facilitating cancer progression.

Currently, little is researched about how miRNA-93-5p functions in BUC. This study firstly predicted its underlying target gene KLF9. Then, the regulation of miRNA-93-5pon KLF9 in BUC was scrutinized. A study reported that KLF9 represses interferon-related signaling to prevent colorectal cancer [22]. miRNA-20a-5p hastens non-small-cell lung cancer cell proliferation by suppressing KLF9 [23]. circPTPRA/miRNA-636/KLF9 is capable of mediating bladder cancer proliferation as clarified by He et al. [24]. However, the potential mechanism of KLF9 in BUC remains to be perfect. Here, KLF9 expression was downregulated in BUC as tested through cell biological experiments. Furthermore, KLF9 overexpression restrained BUC cell migration, proliferation, and invasion and stimulated cell apoptosis in BUC compared with those in the control group, suggesting that KLF9 restrained malignant progression of BUC. Besides, the targeting relationship between miRNA-93-5p and KLF9 was confirmed. Rescue assay proved that miRNA-93-5p inhibited KLF9 expression to exacerbate BUC. These conclusions provide the potential mechanism of KLF9 in BUC, perfect the theory of KLF9 as a cancer regulator, and help for precision medication of BUC. Pathway enrichment analysis of KLF9 uncovered its tight link to the JAK/STAT3 pathway (Supplementary Figure 1A). Western blot suggested that KLF9 overexpression evidently repressed JAK-STAT3-related protein expression, whereas miRNA-93-5p overexpression restored levels of these proteins to the miR-NC+oe-NC level (Supplementary Figure 1B).

All in all, this study proved that miRNA-93-5p deteriorated BUC. We elaborated miRNA-93-5p/KLF9 network in BUC cell processes. The result uncovered the regulation of miRNA-93-5p in BUC cell functions, providing a novel potential therapeutic target.

## Figures and Tables

**Figure 1:** miRNA-93-5p expression is increased in BUC cells. (a) Volcano plot of differential miRNAs in TCGA-BLCA dataset in the normal group and the tumor group. Red refers to upregulated genes, and green refers to downregulated genes. (b) miRNA-93-5p expression in normal samples and tumor samples. Blue boxplot refers to normal samples, and red boxplot refers to tumor samples. (c) qRT-PCR detect the expression of miRNA-93-5p in normal and cancer cells. ^∗^*p* < 0.05.

**Figure 2:** miRNA-93-5p overexpression stimulates BUC cell malignant phenotypes. (a) Transfection efficiency of miRNA-93-5p in RT4 and RT-112 cells in miR-NC and miR-mimic groups. (b) Cell viability in groups. (c) Cell invasive ability in groups (100x). (d) Cell migratory ability in groups (40x). (e) Cell apoptotic rate in groups. ^∗^*p* < 0.05.

**Figure 3:** KLF9 is lowly expressed in BUC cells. (a) Volcano plot of differential mRNAs in a dataset. Red: upregulated; green: downregulated. (b) Venn diagram of predicted target mRNAs of miRNA-93-5p and differentially downregulated mRNAs. Yellow refers to miRTarBase. Orange refers to the TargetScan database. Brown refers to differentially downregulated mRNAs in TCGA-BLCA. Green refers to the miRanda database. Blue refers to the starBase database. Red refers to the miRDB database. (c) Pearson correlation analysis of miRNA-93-5p and candidate genes. (d) Pearson correlation analysis of miRNA-93-5p and KLF9. (e) KLF9 expression in the TCGA-BLCA dataset. Blue refers to normal samples, and red refers to tumor samples. (f, g) KLF9 mRNA and protein expression levels in normal and cancer cells. ^∗^*p* < 0.05.

**Figure 4:** miRNA-93-5p downregulates KLF9 expression. (a) Putative binding sites of miRNA-93-5pon KLF9-WT/KLF9-MUT 3′UTR. (b) Dual-luciferase assay detected luciferase activity of BUC cell line RT4 in miR-NC and miR-mimic groups. (c, d) KLF9 mRNA and protein expression in BUC cell line in miR-NC and miR-mimic groups. ^∗^*p* < 0.05.

**Figure 5:** miRNA-93-5p accelerates BUC through targeting KLF9. (a, b) KLF9 mRNA and protein levels in BUC cell line RT4 upon transfection. (c) Cell proliferation in transfection groups. (d) Cell invasion in transfection groups (100x). (e) Cell invasion in different groups (40x). (f) Cell apoptotic rate in transfection groups. ^∗^*p* < 0.05.

**Table 1:** Cell lines used in the experiments.

Cell line	Type	Num.	Company	Origin
SV-HUC-1	Immortalized human uroepithelial cell line	BNCC100273	BNCC	Shanghai, China
5637	Human BUC cell line	BNCC339635	BNCC	Shanghai, China
RT-112	Human BUC cell line	BNCC338496	BNCC	Shanghai, China
RT4	Human BUC cell line	BNCC341182	BNCC	Shanghai, China
BT-B	Human BUC cell line	BNCC352199	BNCC	Shanghai, China

**Table 2:** qRT-PCR primer sequences.

Gene	Sequence	
miRNA-93-5p	Forward	5′-GCCATGTAAACATCTCGGACTG-3′
	Reverse	5′-CAATGCGTGTGGTGGAGGAG-3′
U6	Forward	5′-GCTTCGGCAGCACATATACTAAAAT-3′
	Reverse	5′-CGCTTCAGAATTTGCGTGTCAT-3′
KLF9	Forward	5′-ACAGTGGCTGTGGGAAAGTC-3′
	Reverse	5′-TCACAAAGCGTTGGCCAGCG-3′
GAPDH	Forward	5′-AGGTCGGTGTGAACGGATTTG-3′
	Reverse	5′-TGTAGACCATGTAGTTGAGGTCA-3′

## Data Availability

The data used to support the findings of this study are included within the article. The data and materials in the current study are available from the corresponding author on reasonable request.

## Supplementary Materials

Supplementary Materials Supplementary Figure 1: JAK/STAT3 pathway mediated by miRNA-93-5p/KLF9.
